The article "Clinical and Laboratory Predictors of Painful Vaso-Occlusive Crisis Among Sickle Cell Disease Patients: A Single-Center Study in Saudi Arabia" was published in 2021. Journal: Cureus.

# Clinical and Laboratory Predictors of Painful Vaso-Occlusive Crisis Among Sickle Cell Disease Patients: A Single-Center Study in Saudi Arabia

**DOI:** 10.7759/cureus.14980

**Published:** 2021-05-12

**Authors:** Ossama Zakaria, Rayan A Buhalim, Fahad Almulhim, Faisal A Al Jabr, Aqeel Alrashid, Mohammed Almutairi

**Affiliations:** 1 Department of Surgery, College of Medicine, Al-Ahsa, SAU; 2 College of Medicine, King Faisal University, Al-Ahsa, SAU

**Keywords:** sickle cell anemia, saudi arabia, vaso-occlusive crisis, parameters, laboratory, profile, sickle cell disease, painful crisis, predictive, markers

## Abstract

Introduction

Vaso-occlusive crisis (VOC) episodes are considered to be the cause of 95% of hospitalizations for sickle cell disease (SCD) patients. The frequency of VOC is significantly associated with higher or lower lactate dehydrogenase levels, higher hemoglobin concentration, higher white blood cell, and neutrophil count, and lower platelet counts. In this study, we highlighted the association and predictors of VOC episodes in Saudi Arabia.

Methods

This is a retrospective observational study that was conducted in a period from January 2018 to December 2019 which included patients who were admitted and treated as sickle cell disease patients were included in this study. Retrieved data included patients' age, sex, and other demographic data items as well as the clinical history of SCD. The patients were divided into two groups. Those patients who developed one or two VOC episodes in the period between 2018-2019 were considered mild in severity and patients who developed three or more VOC episodes in the period between 2018-2019 were categorized as moderate to severe.

Results

A total of ninety-four patients (58 males and 36 females) with a male to female ratio of 1.6 were included in this study. The prevalence of patients who had severe vaso-occlusive crisis was 39.4% while mild-moderate were detected among 60.6% of the patients. It was found that there was no significant difference between the frequency of vaso-occlusive crisis and all the hematological parameters (all p>0.05). It was found that the risk of having vaso-occlusive crisis for those patients who were admitted more than three times was 30 times higher than those patients who were admitted by three times or less [adjusted odds ratio (AOR) = 30.081; 95% confidence interval (CI) = 8.204 - 110.3; p<0.001)].

Conclusion

It was found that those patients who had three times VOC episodes in our studied period are more liable to have frequent episodes in the future which might necessitate urgent intervention for these patients.

## Introduction

Sickle cell disease (SCD) is a hereditary hematological disorder that is inherited in an autosomal recessive manner [1]. It is classified under hemoglobinopathy disorders which are characterized by both intravascular and extravascular hemolysis due to a defect in the hemoglobin molecule of the erythrocytes [2-4]. SCD is caused by a single gene mutation, specifically point mutation, with resultant substitution of the glutamic acid with valine at position six of the beta-globin chain on chromosome 11 [3,5]. SCD can affect multiple organs due to the sickling of erythrocytes and resultant vaso-occlusion, along with hemolytic anemia [6]. Patients with SCD are at risk of various complications, including vaso-occlusive crises, stroke, proliferative retinopathy, acute chest syndrome, splenic atrophy with the consequence of more susceptibility to certain infections, nephropathy, gallstones, osteomyelitis, avascular necrosis (AVN), and more of other systemic complications [2,3,6].

Vaso-occlusive crisis (VOC) episodes are considered to be the cause of 95% of hospitalizations for SCD patients [7]. With certain precipitating factors, the hemoglobin S (HbS) starts to undergo polymerization and change the normal biconcave shape and flexibility of red blood cells (RBCs) into more sickled RBCs. The new sickled erythrocytes are more rigid and have lost their normal flow properties through the microcirculation, with the outcome of erythrocytes being aggregated as well as adhering to the vascular endothelium which causes vaso-occlusion [2,3,8]. This eventually results in ischemic tissue damage and inflammation causing severe pain [9,10]. As a result, VOC manifests as severe pain, especially in the back, joints, and extremities that lasts between three and seven days with the prodromal phase of one to two days [8,11].

In general, the different complications of SCD have their own predictive values. For example, a splenic sequestration crisis has a higher recurrence rate if the spleen size is more than 3 cm, reticulocyte count is greater than 300,000/mm2, and chronic pallor [12]. Moreover, in the case of AVN, the laboratory predictive value for the recurrence is a high steady-state platelet count [13]. However, the frequent VOC are clinical predictors for more symptomatic AVN [14].

In VOC, the frequency of painful crises is significantly associated with higher [15] or lower lactate dehydrogenase levels [16], higher hemoglobin concentration, higher white blood cell and neutrophils count [16,17], and lower platelet counts [18]. It is also significantly correlated with pain-related gene variants [19], hospitalization rates [20], presence of thalassemia [16], and some SCD complications like nephropathy, stroke, and AVN [17]. To our knowledge, there are no studies in regards to clinical and laboratory predictors for painful VOC in Saudi Arabia. Thus, this study is the first to evaluate these predictors thoroughly.

## Materials and methods

Study procedure

This is a retrospective observational study that was conducted in a period from January 2018 to December 2019 for admitted patients in the same period.

This study was conducted from all patients’ records to retrieve their data including sociodemographic data as well as the clinical presentations, hospital course including the laboratory findings, performed surgeries, and comorbidities.

The patients were divided into two groups according to the severity of the VOC in SCD patients defined as mild or moderate to severe as it was used in previous work [17]. Those patients who developed one or two VOC episodes in the period between 2018-2019 year were categorized as mild in severity. Patients who developed three or more VOC episodes in the period between 2018-2019 were categorized as moderate to severe.

Those who are Saudis, have SCD, previously admitted in the ward, males, and females, aged 18 and above were included in this study. However, others were excluded from this study.

Statistical analysis

The descriptive statistics were presented using numbers, percentages mean, and standard deviation, whenever appropriate. Univariate analyses were performed using Fischer Exact test as well as an independent t-test. Multivariate regression analysis was also conducted to determine the effect of the severe Vaso-occlusive crisis where the adjusted odds ratio, as well as 95% confidence interval, were also being reported. A P-value ≤0.05 was considered statistically significant. The data analyses were performed using Statistical Packages for Social Sciences (SPSS) version 21 Armonk, NY: IBM Corporation.

Ethical considerations

Ethical approval was obtained from the ethical committee of the College of Medicine at King Faisal University. Also, consent and approval from the studied setting were obtained before the commencement of the study.

## Results

We analyzed 94 patients who were diagnosed with sickle cell disease. As seen in Table 1, approximately 60% were in the younger age group (≤30 years) with the majority were males (61.7%) and more than half (56.4%) were not married. We further observed 35.1% who were having associated comorbidities. However, 68.1% of the patients were admitted to the hospital three times or less during the last year. Furthermore, the prevalence of patients who had severe vaso-occlusive crisis was 39.4% while mild-moderate ones were detected among 60.6% of the patients. Likewise, the proportion of patients who underwent the operation was 53.2% while the proportion of patients who experienced complications was 68.1%. In addition, all patients took medication for the management of the disease.

**Table 1:** Baseline characteristics of the patients (n=94) SCD: Sickle Cell Disease; ACS: Acute Chest Syndrome.

Study variables	N (%)
Age group	
≤30 years	55 (58.5%)
>30 years	39 (41.5%)
Gender	
Male	58 (61.7%)
Female	36 (38.3%)
Marital status	
Unmarried	53 (56.4%)
Married	41 (43.6%)
Comorbidities	
Yes	33 (35.1%)
No	61 (64.9%)
Frequency of hospitalization	
≤3 times	64 (68.1%)
>3 times	30 (31.9%)
Frequency of vaso-occlusive crisis	
Mild-Moderate (<3 times)	57 (60.6%)
Severe (≥3 times)	37 (39.4%)
Operation	
Yes	50 (53.2%)
No	44 (46.8%)
Medications	
Yes	94 (100%)
No	0
Complications	
Yes	64 (68.1%)
No	30 (31.9%)

Table 2 showed the mean values of different hematological parameters. It was found that the mean values of white blood cells, hemoglobin, platelet, Lactate dehydrogenase (LDH), total bilirubin, and direct bilirubin were 11.4, 9.32, 351.4, 409.2, 36.9, and 22.7, respectively while the mean values of hemoglobin electrophoresis, hemoglobin S, hemoglobin A2, hemoglobin A, and hemoglobin F were 1.85, 64.0, 2.87, 34.3 and 15.6, respectively. Additionally, the mean number of blood transfusions was 3.81.

**Table 2:** Hematological parameters (n=94)

Variables	Mean ± SD
White blood count	11.4 ± 5.77
Hemoglobin	9.32 ± 1.75
Platelet	351.4 ± 439.0
Lactate dehydrogenase	409.2 ± 421.2
Total Bilirubin	36.9 ± 43.8
Direct Bilirubin	22.7 ± 60.8
Hemoglobin Electrophoresis	1.85 ± 0.36
Hemoglobin S	64.0 ± 24.1
Hemoglobin A2	2.87 ± 0.91
Hemoglobin A	34.3 ± 38.4
Hemoglobin F	15.6 ± 10.0
Number of blood transfusion	3.81 ± 2.49

Figure 1 presented the type of procedure done to the patients. It was revealed that the most commonly performed procedure was cholecystectomy (36.2%), followed by splenectomy (12.8%) and hip replacement (3.2%).

**Figure 1:** Type of procedure performed to patients

Figure 2 depicted the prescribed medications to patients. It was found that the most commonly prescribed medication was analgesics (100%), followed by folic acid (95.7%) and narcotics (91.5%).

**Figure 2:** Type of prescribed medications

In Figure 3, the most frequently mentioned complication was a hemolytic crisis (30.9%) and acute chest syndrome (30.9%) followed by gallstone (26.6%) while the least of them was an aplastic crisis (1.1%).

**Figure 3:** Complications

In univariate analysis of the vaso-occlusive crisis, it was revealed that frequency of hospitalization (p<0.001), other procedures (p=0.050), narcotics (p=0.020), hydroxyurea (p=0.045), and avascular necrosis (p<0.001) were the factors associated with vaso-occlusive crisis (Table 3).

**Table 3:** Univariate analysis to determine the factors associated with vaso-occlusive crisis (n=94) § P-value has been calculated using Fischer Exact test. ** Significant at p≤0.05 level.

Factor	Frequency of Vaso-occlusive Crisis		P-value ^§^
	Severe (≥3) N (%) ^(n=37)^	Mild-moderate (<3) N (%) ^(n=57)^	
Age group			
≤30 years	23 (62.2%)	32 (56.1%)	0.669
>30 years	14 (37.8%)	25 (43.9%)	
Gender			
Male	23 (62.2%)	35 (61.4%)	1.000
Female	14 (37.8%)	22 (38.6%)	
Marital status			
Unmarried	23 (62.2%)	30 (52.6%)	0.401
Married	14 (37.8%)	27 (47.4%)	
Comorbidities			
Yes	14 (37.8%)	19 (33.3%)	0.665
No	23 (62.2%)	38 (66.7%)	
Frequency of hospitalization			
≤3 times	11 (29.7%)	53 (93.0%)	<0.001 **
>3 times	26 (70.3%)	04 (07.0%)	
Operation	21 (56.8%)	29 (50.9%)	0.673
Cholecystectomy	15 (40.5%)	19 (33.3%)	0.515
Splenectomy	04 (10.8%)	08 (14.0%)	0.759
Hip replacement	01 (02.7%)	02 (03.5%)	1.000
Other procedures	10 (27.0%)	06 (10.5%)	0.050 **
Narcotics	37 (100%)	49 (86.0%)	0.020 **
Folic Acid	35 (94.6%)	55 (96.5%)	0.645
Hydroxyurea	13 (35.1%)	09 (15.8%)	0.045 **
Complication	27 (73.0%)	37 (64.9%)	0.499
Acute Chest syndrome	10 (27.0%)	19 (33.3%)	0.649
Splenic Sequestration	04 (10.8%)	04 (07.0%)	0.708
Sequestration crisis	0	04 (07.0%)	0.151
Hemolytic crisis	14 (37.8%)	15 (26.3%)	0.260
Aplastic crisis	01 (02.7%)	0	0.394
Gall stone	13 (35.1%)	12 (21.1%)	0.156
Stroke	01 (02.7%)	01 (01.8%)	1.000
Avascular necrosis	08 (21.6%)	0	<0.001 **
Nephropathy	01 (02.7%)	02 (03.5%)	1.000
Osteomyelitis	02 (05.4%)	04 (07.0%)	1.000
Arthritis	01 (02.7%)	01 (01.8%)	1.000
Hypersplenism	03 (08.1%)	08 (14.0%)	0.518

In the comparison between vaso-occlusive crisis and hematological parameters. It was found that there was no significant difference between the frequency of vaso-occlusive crisis and all the hematological parameters (all p>0.05) (Table 4).

**Table 4:** Comparison between vaso-occlusive crisis and hematological parameters (n=94) § P-value has been calculated using Fischer Exact test.  ‡ P-value has been calculated using Independent t-test. ** Significant at p≤0.05 level.

Parameters	Frequency of Vaso-occlusive Crisis		P-value ^‡^
	Severe (≥3) Mean ± SD	Mild-moderate (<3) Mean ± SD	
White blood count	10.8 ± 4.41	11.8 ± 6.57	0.397
Hemoglobin	9.03 ± 1.57	9.52 ± 1.86	0.187
Platelet	412.2 ± 629.0	306.4 ± 206.8	0.269
Lactate dehydrogenase	499.9 ± 447.3	322.0 ± 382.9	0.133
Total Bilirubin	37.2 ± 36.3	36.8 ± 49.4	0.973
Direct Bilirubin	25.6 ± 76.9	20.3 ± 44.2	0.738
Hemoglobin Electrophoresis	1.84 ± 0.37	1.86 ± 0.35	0.775
Hemoglobin S	59.3 ± 23.4	68.0 ± 25.8	0.538
Hemoglobin A2	2.50 ± 0.72	3.10 ± 0.98	0.260
Hemoglobin A	54.4 ± 41.9	24.2 ± 38.2	0.424
Hemoglobin F	18.2 ± 13.8	14.0 ± 7.45	0.489
Number of blood transfusion	4.08 ± 2.45	3.59 ± 2.55	0.470

When conducting multivariate regression analysis to determine the effect of severe vaso-occlusive crisis in relation to the selected baseline characteristics of the patients, we have learned that the risk of having vaso-occlusive crisis for those patients who were admitted more than three times was 30 times higher than those patients who were admitted by three times or less (AOR=30.081; 95% CI=8.204 - 110.3; p<0.001). Other variables included in the model such as other procedures, narcotics, and hydroxyurea were observed to have no significant effect with vaso-occlusive after adjustment to regression model (Table 5).

**Table 5:** Multivariate regression analysis to determine the effect of severe Vaso-occlusive crisis (n=94) AOR: Adjusted Odds Ratio; CI: Confidence Interval. ** Significant at p≤0.05 level.

Factor	AOR	95% CI	P-value
Frequency of hospitalization			
≤3 times	Ref		
>3 times	30.081	8.204 – 110.3	<0.001 **
Other procedures			
Yes	0.283	0.039 – 2.053	0.212
No	Ref		
Narcotics			
Yes	2.990	0.627 – 14.270	0.170
No	Ref		
Hydroxyurea			
Yes	3.411	0.738 – 15.775	0.116
No	Ref		

## Discussion

Sickle cell disease (SCD) is one the most prevalent hematological diseases in Saudi Arabia [21], in which it is associated with several complications such as vaso-occlusive crises, avascular necrosis (AVN), gallstones, acute chest syndrome, splenic atrophy, and others [2,3,6]. Several studies showed that various clinical and laboratory findings could be associated with the frequency of their complications. However, they were not conducted in Saudi Arabia. Thus, in this study, we highlighted this issue to make it a base for further studies.

As demonstrated in Table 1, the majority of our patients were less than 30 years of age, which is similar to a previous study from the literature [17]. As observed in Table 3, the most common surgical operation for SCD patients is cholecystectomy, which is consistent with a previous study [22]. This is because these patients tend to have chronic hemolysis which causes the formation of pigment gall stones and necessitates cholecystectomy. However, a previous study stated that most of the included patients were hospitalized less than three times which is similar to our findings in Table 1. We also support the findings in which hemolytic crisis is the most common complication among SCD patients [23].

As demonstrated in Table 3, it is revealed in our study that several factors are significantly associated with the vaso-occlusive crisis severity such as increased number of hospitalizations, number of the administered narcotic analgesia, taking hydroxyurea, and AVN. Similarly, a previously conducted study supports our findings which is, an increased number of vaso-occlusive events is significantly associated with an increased number of hospitalizations as well as AVN [17], and another study supports the finding of the AVN [14]. This similarity of the results between the studies suggests serious consideration of these factors as predictors of further vaso-occlusive attacks. Moreover, further studies are needed to confirm and explore the reason behind these findings and to put the required preventive measures.

Previous studies have shown that there are several significant predictors for the severity of the vaso-occlusive crisis such as higher white blood cell count, higher lactate dehydrogenase, higher hemoglobin level, higher steady platelet count, alpha-thalassemia trait, hemoglobin SS phenotype [8,15,17,18,20]. On the other hand, there was no significant difference between the frequency of vaso-occlusive crisis and all the hematological parameters included in our study as seen in Table 2. Furthermore, another study showed similar results to our study [14].

Our study has significantly shown that patients who have been admitted more than three times have a 30 times higher risk for severe vaso-occlusive crisis compared to patients who were admitted three times or less. Also, one study showed that patients with frequent hospital readmissions because of vaso-occlusive crisis have poor outcomes, prognosis, and demand more care and monitoring [7].

Limitations

Besides the limitation of being a low sample size study, the authors recommend that future prospective studies should be conducted to enhance the quality of data.

## Conclusions

Despite the authors could not find a significant association between VOC episodes and the hematological parameters, the study concluded that those patients who had three times VOC episodes are more liable to have frequent episodes in the future. This study supports the earlier use of hydroxyurea to avoid such complications of frequent crises. However, a larger sample size with prospective studies is recommended to be done in the future.
